# Research on Intelligent Solution of Service Industry Supply Chain Network Optimization Based on Genetic Algorithm

This article has been retracted.

**DOI:** 10.1155/2021/9429872

**Published:** 2021-08-19

**Authors:** Yixin Zhou, Zhen Guo

**Affiliations:** ^1^School of Business Economics, Shanghai Business School, Shanghai 201400, China; ^2^School of Economics, Harbin University of Commerce, Harbin 150000, Heilongjiang, China

## Abstract

With the advent of the era of big data (BD), people”s living standards and lifestyle have been greatly changed, and people's requirements for the service level of the service industry are becoming higher and higher. The personalized needs of customers and private customization have become the hot issues of current research. The service industry is the core enterprise of the service industry. Optimizing the service industry supply network and reasonably allocating the tasks are the focus of the research at home and abroad. Under the background of BD, this paper takes the optimization of service industry supply network as the research object and studies the task allocation optimization of service industry supply network based on the analysis of customers' personalized demand and user behavior. This paper optimizes the supply chain network of service industry based on genetic algorithm (GA), designs genetic operator, effectively avoids the premature of the algorithm, and improves the operation efficiency of the algorithm. The experimental results show that when *m* = 8 and *n* = 40, the average running time of the improved GA is 54.1 s. The network optimization running time of the algorithm used in this paper is very fast, and the stability is also higher.

## 1. Introduction

With the increasing competition in the world market, competition is no longer a competition between enterprises, but a competition between supply chains. The basis of competition between supply chains is the competition of supply chain networks [1–3]. Efficient supply chain network can not only reduce the operating costs of enterprises, but also respond to market demand quickly, reduce operational risks, and improve the overall competitiveness. But at present, with the expansion of enterprise scale, the hub distribution center of enterprise supply chain network is also expanding rapidly, seizing the market share, resulting in many hub locations design unreasonable [4]. Moreover, due to the straight-line organization and management mode implemented by most enterprises in China, the repeated transportation between distribution centers within enterprise groups is serious, the inventory is too large, the market response speed is slow, and the profitability is poor [5]. Supply chain refers to a functional network chain structure that centers around the core enterprise, starting from supporting parts, making intermediate products and final products, and finally sending products to consumers by the sales network, connecting suppliers, manufacturers, distributors, and end users as a whole. The business philosophy of supply chain management is to seek the overall optimization of the supply chain from the perspective of consumers and through the cooperation between enterprises.

Supply chain refers to the chain structure or network related to the production and distribution of raw material suppliers, producers, wholesalers, retailers, and end users [6]. The relevant processes of supply chain include procurement, production, value-added, distribution, information exchange, and exchange between different business entities, which has a balanced effect [7]. An enterprise is a node, and there is an exchange of interests between nodes and node enterprises. Supply chain usually has the characteristics of complex, dynamic, and user-oriented demand [8, 9]. However, in today's market, supply chain has other functions, such as rapid response, function integration, goal setting management, modernization, and enterprise network and information electronics [10]. Supply chain management refers to all kinds of activities and processes that plan, coordinate, operate, control, and optimize the whole supply chain system. Its goal is to deliver the right products needed by customers to the right place at the right time according to the right quantity, quality, and status and to minimize the total cost of this process. Obviously, supply chain management is a kind of management mode embodying the idea of integration and coordination.

Based on this, this paper proposes an improved genetic operator algorithm to study the optimization of service supply chain network. This paper first introduces the basic concepts of BD and supply chain and then improves the traditional genetic operator, aiming at the existing multilevel logistics network, which does not fully consider the customer's potential interest demand. Under the background of BD, this paper puts forward a design method based on the analysis of customer's network score to the distributor, predicts the potential interest factors of customers, and introduces the prediction results into the design method of multilevel logistics network optimization. The experimental results show that the improved GA used in this paper has fast average running speed and good stability, and customers' evaluation of logistics network is very high. In the information integration mode of supply chain management, enterprises should choose supply chain partners as the information cooperation objects as far as possible to implement supply chain informatization. This is because the fundamental goal of enterprises is to maximize their own profits, and the realization of this goal is achieved by well meeting the needs of downstream enterprises. In this process, it must also rely on the supply of upstream enterprises.

## 2. Overview of GA and Supply Chain Network Modeling

### 2.1. Concept of GA

GA is a random search method developed from the evolution law of biology in the biological world, which is the genetic mechanism of survival of the messenger and survival of the fittest proposed by Darwin. The main function of GA is to automatically find and orient the adjusted search space and use the probability optimization technology that can adjust the search direction accordingly. At present, GA has been widely used in management, development, program planning, and other fields. Besides, because genetic algorithm canno't deal with the parameters of the problem space directly, the problem to be solved must be expressed as chromosome or individual in the genetic space by coding. This conversion operation is called encoding. The following three criteria are often used to evaluate coding strategies: (a) completeness: all points (candidate solutions) in the problem space can be represented as points (chromosomes) in the GA space; (b) soundness: chromosomes in GA space can correspond to candidate solutions in all problem spaces; (c) nonredundancy: chromosomes and candidate solutions correspond one by one.

The basic idea of GA is expressed in the language of an algorithm: at the beginning of the calculation process, some individuals or populations are started randomly, and the fitness function of each individual is calculated at the same time. Then the next generation is created according to the first generation that satisfies the adaptive function. If the optimization criteria are not met at this time, a new round of calculation will be started. Only individuals that meet the fitness selection can produce the next generation, while the father generation needs gene recombination to produce offspring. All races are created by accident. Then, according to the number of offspring or population, the gene is recalculated and transferred to the next generation to form a new generation. Repeat the process until the optimization criteria are met.

### 2.2. Supply Chain Modeling Based on Improved GA

The content of GA optimization is based on the ability of each individual in the group. Adaptive people tend to engage in frequent activities such as selection and transportation and eventually find a solution to the problem. Fitness function is the standard to evaluate the quality of individuals in a population, and it is the only basis to imitate natural selection. Therefore, the selection of fitness function directly affects the speed of GA change and the best solution. In genetic algorithm, individuals in the initial population are randomly generated. Generally speaking, the initial group can be set as follows: (a) according to the inherent knowledge of the problem, try to grasp the distribution range of the space occupied by the optimal solution in the whole problem space, and then set the initial group within this distribution range; (b) firstly, a certain number of individuals are randomly generated, and then the best individuals are selected and added to the initial population. This process iterates until the number of individuals in the initial population reaches a predetermined size.

Since the objective function of the distribution network optimization model based on inventory control is to find the minimum total cost of the system, the minimum form of fitness function is used to map the objective function to the fitness function.

(1) $$\begin{array}{c} F\left(x\right)=\left\{\begin{array}{cc} C_{\max}-f\left(x\right), & f\left(x\right)<C_{\max},\\ 0, & \text{Other information.} \end{array}\right. \end{array}$$

Among them, *F*(*x*) is the fitness function, *f*(*x*) is the objective function, *C*_max_ is the appropriate relatively large number, and the value is the maximum objective function value in the current or recent generations. The recombination of biological genetic genes (plus mutation) plays a central role in the process of biological evolution in nature. Similarly, the crossover operator of genetic operation plays a key role in genetic algorithm. The so-called crossover refers to the operation of replacing and reorganizing part of the structure of two parent individuals to generate new individuals. Through crossover, the search ability of genetic algorithm can be greatly improved.

The roulette selection strategy based on fitness ratio is often used in basic GA to select subindividuals. Although the implementation is simple, it is easy to cause premature convergence and slow search in the later stage. In this paper, the selection operator accepts the nonlinear identification option and uses a nonlinear function to map the queue number to the expected probability. Population *P*={*a*_1_, *a*_2_, ⋯*a*_*n*_} was ranked according to the fitness level, *f*(*a*_1_) ≥ *f*(*a*_2_) ≥ ⋯*f*(*a*_*n*_). Using the nonlinear normalized geometric ranking function, the selection probability of individual *i* is as follows:

(2) $$\begin{array}{c} \left\{\begin{array}{c} P\left(i\right)=q^{\prime }{\left(1-q\right)}^{r-1},\\ q^{\prime }=\frac{q}{1-{\left(1-q\right)}^{n}}. \end{array}\right. \end{array}$$

Among them, *q*′ is the best individual selection probability, *r* is the individual sequence number, and *n* is the population size.

Because the network optimization model based on inventory control has constraint conditions, when solving the optimization constraint problem, GA usually transforms the constraint condition into unconstrained optimization problem, and the penalty function method is often used. If the square term of the constraint is used as the penalty function, then the penalty function of the constraint is

(3) $$\begin{array}{c} P_{x}=p{\sum_{i=1}^{m}\left(\sqrt{\frac{2o_{i}}{h_{i}}\sum_{j=1}^{n}\mu_{j}X_{ij}}+\Phi^{-1}\left(\alpha_{i}\right)\sqrt{L_{i}\sum_{j=1}^{n}\delta_{j}^{2}X_{ij}-B_{i}}\right)}^{2}, \end{array}$$

where *p* is the penalty function.

When the fitness of the optimal individual reaches a given threshold, or the fitness of the optimal individual and the population no longer rises, or the number of iterations reaches the preset algebra, the algorithm stops. The default algebra is generally set to 100–500 generations.

## 3. Experimental Background and Design

With the economic development in the 21st century, global economic growth and modern science and technology have become more and more competitive. How to meet the needs of customers, increase market share, and reduce costs to profit is the main challenge faced by enterprises. In this context, the competition between traditional enterprises has gradually shifted to the competition between supply chains, and supply chain management has become an important means to obtain competitive advantages in the process of enterprise development. Therefore, in the era of BD, according to a large number of data such as browsing data, location data, social data, and personal information, we can analyze and mine the potential interests, behavior rules, and decision-making factors of customers. And according to the analysis of customer data results to improve the corresponding service capabilities of enterprises, so as to provide better services for customers, will improve the competitiveness of enterprises in the future and is conducive to the long-term and stable development of enterprises. Genetic algorithm is a general algorithm to solve the search problem, which can be used for all kinds of general problems. The common characteristics of search algorithms are as follows: firstly, a group of candidate solutions are formed; the fitness of these candidate solutions is calculated according to some adaptive conditions; according to the fitness, some candidate solutions are reserved and others are abandoned; some operations are performed on the reserved candidate solutions to generate new candidate solutions.

In this paper, firstly, the relevant theoretical methods, connotation characteristics, and structure of BD analysis and mining technology are described in detail. In the context of BD, this paper studies the theory of customer's personal needs and user behavior rules, as well as customer's online information and location information to analyze potential needs and behavior rules. Secondly, it analyzes the impact of customer's personal demand on logistics supply chain network. The basic theory and model of logistics supply network and logistics service supply chain are elaborated in detail. Finally, an improved genetic operator algorithm is proposed to solve the optimization problem of logistics supply network considering customers' personalized demand, and the prediction results are introduced into the design model of multilevel logistics network optimization. The simulation results show that the decision-making method of choosing different customer needs under different circumstances is an effective and feasible method to improve the service level of logistics network. Because the overall search strategy and optimization search method of genetic algorithm do not depend on gradient information or other auxiliary knowledge, but only need the objective function and the corresponding fitness function that affect the search direction, genetic algorithm provides a general framework for solving complex system problems, which does not depend on the specific domain of the problem. It has strong robustness to the types of problems. Its application fields include function optimization, combinatorial optimization, and job shop scheduling.

## 4. Discussion

### 4.1. Data Set Preparation and Experimental Parameter Setting

In the case of BD, all sales-related information can predict product sales based on customer click, browse time, shopping cart, and review data. If the click-through rate of a product has soared recently, the related product is also the latest hot selling product, so there must be some relationship between the click-through rate and the sales volume. This paper focuses on the relationship between the reaction speed of the model and the number of iterations to predict the sales volume. If one more customer click is added according to the real-time characteristics of BD, the data will be continuously recorded to predict the accurate time of customers. Suppose that the sales volume is *m*, the click-through rate and browse time are A and B, respectively. Select the most recent user click information, and then click the selected one as 1. Otherwise, it is 0. If the browsing time exceeds 30 s, it is 1. Otherwise, it is 0. In the purchase result, the purchase is 1 and the nonpurchase is 0. The data is shown in Table 1.

The model is established in accordance with the following assumptions:

1. Product quality and category differences are not taken into account.
2. A distribution point can serve multiple customers, but a customer can only accept the service of one distribution node.
3. The customer's location data is known.

The experimental equipment of this experiment is Windows, and the software is MATLAB. The experimental parameters are shown in Table 2.

### 4.2. Comparison of Optimization Results between Improved GA and Basic GA

Suppose the distribution network has a product factory, *m* alternative distribution centers, and *n* independent distribution points. Considering the establishment of a distribution center, there are some choices in *M* candidate points, which are responsible for the distribution of goods to the service distribution points in the jurisdiction, thus forming a typical multisource transfer point distribution network, the goal of which is to minimize the total cost of the system.

Through the simulation experiment, the improved GA and the basic GA are repeated 20 times for comparative analysis. The number of individuals in the initial population is 30, and the evolutionary generation is 400 generations. Through the calculation of problems of different scales, the comparison between the improved GA and the basic GA is shown in Figure 1.

According to the data in Figure 1, under the same parameter settings, the operation speed of the improved GA is faster than that of the traditional GA, especially for large-scale problems. When *m* = 8 and *N* = 40, the average running time of the improved GA is 54.1 s, while the average running time of the traditional GA is 97.9 s. It can be seen that the improved GA greatly saves the running time of the algorithm.

According to the data in Figure 2, it can be seen that, under the same parameter setting, the average iteration time of the improved GA is less than that of the traditional GA, and the convergence is good and the stability is strong. When *m* = 8 and *n* = 40, the average operation iteration time of the improved GA is 120, while the average operation time of the traditional GA is 224. The average iteration time of the improved GA is half of that of the traditional GA. The results show that the improved GA has a very good effect on the optimization of service supply chain network.

Finally, this paper analyzes the service level, payment convenience, price, and evaluation and distribution integrity of suppliers. The higher the score value is, the higher the corresponding level is. 1 represents the lowest service level and price, and 5 is the highest score. However, due to the limited space of the article, some customers' main personalized requirements are selected. Customer requirements and supplier rating are shown in Figure 3.

According to the data in Figure 3, the score of service level is 4.5, the score of payment convenience is 4.5, and the score of price, evaluation, and distribution integrity is 5. The overall score is relatively high. The experimental results also show that the supply chain designed by the improved GA can meet some personalized needs of customers, and the optimized supply chain of service industry makes customers very satisfied.

The programming of genetic algorithm is very complex. Firstly, we need to encode the problem and decode the problem after finding the optimal solution. In addition, the implementation of the three operators also has many parameters, such as crossover rate and mutation rate, and the selection of these parameters seriously affects the quality of the solution, but at present, the selection of these parameters mostly depends on experience. The feedback information of the network is not used in time, so the search speed of the algorithm is relatively slow, and it needs more training time to get more accurate solutions.

### 4.3. Network Optimization Strategy

According to the strategy of network optimization, it should be analyzed from five aspects: customer service level, facility location strategy, inventory decision-making strategy, transportation decision-making strategy, integrated location, and the relationship between inventory and transportation.

#### 4.3.1. Customer Service Level

In the distribution network, improving customer service standards in the distribution network will also increase the system cost. A certain level of customer service is always supported by a certain cost. Compared with any other traditional transportation company, the level of customer service provided by the company has a greater impact on the distribution network optimization. Because of the low cost of storage and storage in the enterprise area, the goods can be stored at low cost. On the contrary, the service level is high. However, with the improvement of service level, the cost of distribution network will increase rapidly. Therefore, the premise of distribution network is to determine the level of customer service.

#### 4.3.2. Facility Location Strategy

Distribution network is a kind of network system, including not only the physical network composed of distribution lines and distribution nodes, but also the virtual network composed of computers and communication systems. For distribution network utility, the operation and transportation costs of distribution network equipment are low because the location of distribution network equipment takes into account the number of distribution equipment and the optimal distribution location in the specified or uncertain distribution area according to the conditions of nodes. The core of enterprise location strategy is to find the lowest cost allocation plan. Site selection involves many factors; transportation cost and efficiency are important factors to determine site selection. The site selection in the distribution network is a huge permanent investment institution, logistics center, or distribution center. If the wrong location is detected, it will lead to great loss. The transfer process and cost of all products must be considered when formulating the environmental strategy of the plant through different channels to meet customer needs. For example, customers can be provided directly in factories or indirectly in factories and intermediate units, which will affect customer service standards and service costs.

#### 4.3.3. Inventory Decision Strategy

Inventory decision is the choice of material management and control methods. There are many commodity management strategies in the order. According to whether the test cycle is constant or variable, the test cycle can be divided into a series of test methods and periodic test methods. The ongoing test strategy is divided into order quantity, order point strategy, order point, and maximum control strategy. The current test strategy includes fixed order quantity policy and large quantity policy. Interest in inventory management can be divided into certainty, arbitrariness, and transparency. For example, the factory's demand for raw materials is usually correct, but the demand for goods in sales is usually random or fuzzy.

#### 4.3.4. Transportation Decision Strategy

Transportation decision includes transportation mode selection, transportation collection, and transportation options. The production flow between the two locations can be carried out by a variety of transport modes, each of which has certain limitations in terms of transport capacity and availability. Route selection has a significant impact on transportation costs. Although a route saves less transportation costs, the total cost can be greatly reduced due to the longer available time. Therefore, the enterprise should develop an effective transportation system based on the comprehensive plan and reasonably select the means of transportation, transportation route, and transportation route.

#### 4.3.5. Integrated Location, Inventory, and Transportation Strategy

Facility location, inventory decision, and transportation decision affect each other. The location and function of facilities determine the basic structure of distribution network, which is directly related to the transportation distance and transportation cost of products, and the selection of transportation route and mode also affects the level of the company. Therefore, in the optimization of distribution network, the integration of location, counting, and transportation can be considered to further improve the level of distribution network optimization. The distribution center provides goods distribution services to customers. Now we need to choose the appropriate location of the distribution center (a certain number of locations) or the appropriate number and location of the distribution center (the number of locations and the location are optimized at the same time). The goal is to meet the needs of customers, and it can achieve the goal of shortest distance and minimum logistics cost under certain constraints.

## 5. Conclusions

With the continuous development of BD, people will produce a lot of data when they buy things, and enterprises can use these data to analyze the needs of customers, which can also accelerate the progress of the times. This paper first studies the background of competition among enterprises and then proposes an improved genetic operator algorithm to study the optimization of service supply chain network. Compared with the traditional GA, the experimental results show that the improved GA has faster running speed, better stability, and better convergence. Finally, the improved GA is applied to the supply chain of service industry, and the customer satisfaction is very high, which proves the feasibility and effectiveness of the model and algorithm.

## Figures and Tables

**Figure 1:** Comparative analysis of average running time of two algorithms.

**Figure 2:** Comparative analysis of average iteration times of two algorithms.

**Figure 3:** Evaluation table of logistics network service system.

**Table 1:** Customer's experimental data.

Click-through rate A	Browse time B	Purchase m
1	1	1
1	0	1
1	0	1
0	0	0
1	1	1
1	1	1
1	1	0
1	0	0

**Table 2:** Experimental parameters.

Parameter name	Basic genetic algorithm	Improved genetic algorithm
Coding method	Binary coding	Binary and symbol coding
Selection operator	Roulette	Nonlinear sorting selection
Crossover operator	Single point crossing (0.75)	Two-point crossing (0.9,0.75,0.6)
Mutation operator	Single point crossing (0.04)	Single point crossing (0.1,0.04,0.01)

## Data Availability

The data underlying the results presented in the study are available within the manuscript.
